The article "The Effects of Foot Reflexology for Smoking Cessation on Brain Activities with Functional Magnetic Resonance Imaging (fMRI): A Pilot Study" was published in 2022. Journal: Evid Based Complement Alternat Med.

# The Effects of Foot Reflexology for Smoking Cessation on Brain Activities with Functional Magnetic Resonance Imaging (fMRI): A Pilot Study

**DOI:** 10.1155/2022/1727479

**Published:** 2022-07-09

**Authors:** Pisit Wattanaruangkowit, Sombat Muengtaweepongsa, Mondha Kengganpanich, Tharadol Kengganpanich

**Affiliations:** ^1^Department of Radiology, Faculty of Medicine, Thammasat University, Pathum Thani 12120, Thailand; ^2^Center of Excellence in Stroke, Faculty of Medicine, Thammasat University, Pathum Thani 12120, Thailand; ^3^Department of Health Education and Behavioral Sciences, Faculty of Public Health, Mahidol University, Bangkok 10400, Thailand

## Abstract

**Background:**

Foot reflexology is a treatment with the hypothesis that such massage stimulation on the feet may cause a therapeutic effect which should be helpful for smoking cessation. However, its mechanism of action in the brain of smoking people remains unknown. Functional magnetic resonance imaging (fMRI) is helpful for real-time brain activity detection. We aim to compare the brain activity effects of foot reflexology with fMRI between smoking and nonsmoking subjects.

**Materials and Methods:**

We divided participants into experimental (smokers) and control groups (nonsmokers). Both groups received similar foot reflexology under the fMRI examination. Then, we compared the mean response score in each brain area before and after foot stimulation among groups and between groups.

**Results:**

Five nonsmokers and fifteen smokers had completed the study. All participants were right-handed males, with a mean age of 38.6 years. The fMRI brain response in the areas correlated with foot stimulation, including the precentral gyrus of the frontal lobe and the postcentral gyrus of the parietal lobe, was present for all participants. The fMRI response outside the correlated area, including other parts of the frontal and parietal lobes, the temporal and occipital cortices, and the thalamus, was also found in all participants, but was not consistent.

**Conclusions:**

The fMRI of the brain is feasible and safe for demonstrating foot reflexology reactions. The response signal outside the correlated motor-sensory cortical area with foot reflexology may have clinical significance and may be helpful for smoking cessation. We suggest conducting a large-scale, randomized controlled trial to confirm these findings.

## 1. Introduction

Foot reflexology is a system of massage used to activate homeostasis, based on the theory that reflex points exist on the feet linked to every part of the body. It helps relieve pain and anxiety and improve sleep quality in patients with many diseases [1–3]. However, the mechanism of the reflexology is still uncertain [4]. Some previous studies suggested that foot massage at reflex points despite unilateral sole may activate the brain, as demonstrated in bilateral electroencephalographic changes [5, 6]. The reflexological stimulation at the reflex points on the soles activates the correlated somatosensory cortex and their reflex areas in the brain. Functional magnetic resonance imaging (fMRI) can demonstrate these significant effects [7].

fMRI brain is generally used for relevant sensorimotor task performance [8]. The most often used technique to detect the functional changes in the brain is blood oxygenation level-dependent (BOLD) fMRI [9]. Neurologists used BOLD fMRI to diagnose many neurological diseases, including sensory disorders [10]. fMRI brain could demonstrate the outside corresponded somatosensory activation during acupuncture [11]. A few previous studies reported the use of fMRI to detect brain activity in reflexology [7, 12]. A reflexologic expert recommended using fMRI as a surrogate marker of brain activity in patients treated with reflexology [13].

The World Health Organization stated that cigarette smoking had become one of the biggest public health threats the world has ever faced [14]. Less than five percent of smokers can quit without professional assistance [15]. Family and social support are the keys to success for smoking cessation [16]. Foot reflexology has been used in Thailand's tobacco control program for more than ten years. The community-based tobacco control program is becoming more and more widely used to help quit smoking in public health facilities, especially at the local level, including health-promoting hospitals. The successful smoking cessation rate rose to almost 50% with foot reflexology stimulation [17].

We conducted a pilot study to compare the brain activity effects of foot reflexology with fMRI between smoking and nonsmoking subjects.

## 2. Methods

This study is a double-blinded (participants and interpretation) clinical trial. We divided participants into experimental (smokers) and control groups (nonsmokers). Both groups do not know which group they are in (experimental or control group). In the fMRI test, the investigators will perform tests without knowing which group is the experimental or control group. The voluntary participants in the experimental group have had a habit of smoking regularly for at least one year. The study followed through in agreement with the Declaration of Helsinki (2008) of the World Medical Association. The Ethical Review Committee for Human Research, Faculty of Public Health, Mahidol University, approved the study (EC approval number: MOPH-2019-022, issued date: 30 Jan 2020).

The inclusion criteria were as follows: male, aged 20 years and over; the experimental group who were smokers, being a daily smoker who can either smoke the commercial or the domestic cigarette; the control group was nonsmokers; willing to give consent to study. The exclusion criteria were as follows: taking drugs affecting the central nervous system.

We performed the reflexological stimulation under the fMRI examination, where researchers applied the pressure with the right and left thumbs, respectively. Both groups received three plantar reflexological stimulation points (used to help quit smoking). Each point took 45 seconds for pressure application. We took 45-second breaks before the beginning of another pressure application on the same foot until the completion of all three points. Then, we switched the reflexological performance to the other foot. The total duration of the reflexological stimulation was approximately 10 minutes per participant.

The three massage points used in this study include the following (Figure 1):

- Above the hallux next to the toe index finger (area number 1)
- Inside of the hallux attached to the toe index finger (area number 2)
- The outer squares, both the top and bottom of the hallux (area number 3)

For quality control, only one reflexologist gave a treatment to prevent discrepancies between individuals (interpersonal error) on each day of data collection. The reflexologist gave a treatment to no more than five participants a day to prevent any individual discrepancies (intrapersonal error).

All fMRI measurements were performed using a Siemens MAGNETOM Skyra 3.0 Tesla scanner, high-resolution 3D T1 resolution, and an MPRAGE sequence-weighted structural image with a repetition time of (TR) = 1900 ms, echo time (TE) = 2.30 ms, field of view (FOV) = 230 mm, and 0.8 mm slice thickness for rapidly acquiring images. Echo planar imaging (EPI) was defined at TR = 3000 ms, TE = 30 ms, FOV 200 mm, 5.0 mm slice thickness, and spatial distortion of EPI images was reduced using gradient field mapping; TR = 737 ms, TE = 4.92 ms, FOV = 320 mm, and 3.0 mm slice thickness were set, as shown in Table 1.

We collected demographic data and measured carbon monoxide in breath with a smokerlyzer dryer. We used syngo.via workstation software version VB30 for reading fMRI results.

The fMRI response signal was labeled as intense, positive, and negative, giving a score of two, one, and zero, respectively. We compared the mean response score in each brain area before and after foot stimulation among groups and between groups, using the *t*-test. A value of *p* < 0.05 was considered statistically significant.

## 3. Results

Among the 22 participants, we assigned six nonsmokers as a control group. We excluded one in the control group due to the low-quality fMRI resulting from currently taking anxiolytic drugs. Among the remaining 16 smokers assigned to the experimental group, one had a claustrophobic condition and refused to continue testing with MRI. Finally, five nonsmokers in the control group and 15 smokers in the experimental group remained for the study.

All participants in this study were male and right-handed. The left hemisphere was supposed to be dominant in all participants. The mean age was 38.6 years (37.4 years in the experimental group and 38.8 years in the control group). One participant in the experimental group had hypertension. In comparison, two in the control group had hypertension and diabetes.

Table 2 shows the demographic data. According to the inclusion criteria, fifteen smokers in the experimental group had smoked for at least one year. Among the 15 smokers, five smoked domestic cigarettes (No. 17–21), and the rest smoked commercial ones (No. 7–16). The smoking duration ranged from 6 to 24 years averaging 16.2 years (standard deviation of 4.1 years). The number of cigarettes used per day ranged from 5 to 40 with an average of 21.9 (standard deviation of 10.7). Average carbon monoxide in breath ranged from 2 to 24 parts per million (ppm) with an average of 9.7.

When the ipsilateral foot gets massaged, the contralateral correlated cortex, such as the precentral gyrus of the frontal lobe and the postcentral gyrus of the parietal lobe (pre-and post-CG), basically expresses a present signal in the fMRI. The fMRI of the brain response in the area correlated with foot stimulation, including the precentral and postcentral gyri (pre-and post-CG), became intense or present for all participants (Figures 2(a), 2(b), and 3(a)). The signals became intense only at the right postcentral gyrus (sensory area) during left foot stimulation in 13 participants (Table 3). In comparison, the signals became intense during right foot stimulation at the left postcentral gyrus in seven participants (Table 4). We found the response outside the correlated pre- and post-CG, including other parts of the frontal cortex outside the precentral gyrus (Figures 2(c) and 3(b)), other parts of the parietal cortex outside the postcentral gyrus, occipital and temporal cortex, and thalamus, bilaterally (Tables 3 and 4). The fMRI response outside the correlated area in the cerebral hemisphere may lead to therapeutic effects.

## 4. Discussion

To the best of our knowledge, our study is the third report about the manifestations of the fMRI brain with foot reflexological stimulation [7, 12]. We find the activation signals outside the corresponding motor and sensory cortices, including the contralateral frontal, parietal, occipital, temporal cortices, and the thalamus with fMRI. The activation signals are inconsistent and various. Other brain reactions rather than the corresponding foot sensory areas detected by fMRI may imply that foot reflexology may affect other brain parts outside its motor and sensory territories. These fMRI manifestations are similar in both smokers and nonsmokers. Therefore, we cannot conclude whether these findings are positive phenomena for smoking cessation. The most well-known effects of foot reflexology are relaxation and pain relief [18]. We also do not know whether the positive results of foot reflexology on smoking cessation are its indirect consequences of relaxation.

The success rate of smoking cessation with bupropion, a standard medical treatment, is less than 50% [19]. The factors associated with successful smoking cessation are various [20]. Physicians usually provide patients with multimodal approaches to help them achieve absolute smoking cessation [21]. The successful smoking cessation rate of almost 50% with foot reflexology in a previous study is comparable to bupropion treatment but is much less expensive [17]. However, the mechanism of action from foot reflexology to the brain remains uncertain.

Due to lacking scientific evidence and unexplained mechanism of action, reflexology remains a nonstandard treatment. Healthcare professionals do not recommend reflexology for treating any medical diseases. Patients seeking reflexology may get delayed from the appropriate medical treatment. However, the relaxation effects and direct harmlessness are the advantages of reflexology. It is an excellent reason to apply reflexology in health promotion or disease prevention [22]. Due to its safety, reflexology has become an alternative treatment for pain relief and comfort during labor [23].

The limitations of our study include a small sample size, lacking smoking cessation outcomes, and no sham reflexology for comparison. The prospective randomized control trial of foot reflexology comparison with sham for smoking cessation programs using fMRI as a surrogate marker is suggested for further studies.

In conclusion, the fMRI of the brain is feasible and safe for demonstrating foot reflexology reactions. The response signal outside the correlated motor-sensory cortical area with foot reflexology may have clinical significance and may be helpful for smoking cessation. We suggest conducting a large-scale, randomized controlled trial to confirm these findings.

## Figures and Tables

**Figure 1:** Three massage points.

**Figure 2:** A 31-year-old smoking man. During massage on the left foot; intense signal at the right postcentral gyrus in B (red arrow), the present signal at precentral and postcentral gyri in A (green arrows), and the bilateral frontal lobes in C (blue arrows).

**Figure 3:** A 29-year-old nonsmoking man. During massage on the right foot; intense signal at the left precentral gyrus in A (red arrow), and the present signal at the left frontal lobe in B (blue arrow).

**Table 1:** The details of the MRI machine.

	TR (ms)	TE (ms)	Slice thickness	FOV (mm)	Acquisition matrix	Recon voxel size (mm)
MPRAGE (magnetization-prepared rapid gradient-echo)	1900	2.30	0.8	230	288 × 288	0.8 × 0.8 × 0.8
EPI (echo planar imaging)	3000	30	5.0	200	88 × 88	2.3 × 2.3 × 5.0
Gradient field mapping	737	4.92	3.0	320	64 × 64	5.0 × 5.0 × 3.0

**Table 2:** Demographic data.

No.	Age (years)	Underlying diseases	Smoking history	Type of cigarette	Smoking duration	Smoking intensity (cigarettes/day)	Carbon monoxide (ppm)
1	29	—	Nonsmoker	—	—	—	—
3	25	—	Nonsmoker	—	—	—	—
4	60	Hypertension	Nonsmoker	—	—	—	—
5	52	—	Nonsmoker	—	—	—	—
6	43	—	Nonsmoker	—	—	—	—
7	39	—	Smoker	Commercial cigarettes	24	5	3
8	59	Hypertension	Smoker	Commercial cigarettes	35	10	12
9	26	—	Smoker	Commercial cigarettes	12	5–6	2
10	25	—	Smoker	Commercial cigarettes	5	1–10	11
11	29	—	Smoker	Commercial cigarettes	14	1–2	2
12	30	—	Smoker	Commercial cigarettes	12	7	2
13	35	—	Smoker	Commercial cigarettes	20	10	6
14	25	—	Smoker	Commercial cigarettes	10	20	7
15	32	—	Smoker	Commercial cigarettes	12	10	14
16	43	Hypertension	Smoker	Commercial cigarettes	39	10	9
17	54	—	Smoker	Domestic cigarettes	33	>10	17
18	50	—	Smoker	Domestic cigarettes	34	20	24
19	38	—	Smoker	Domestic cigarettes	25	20	14
20	40	—	Smoker	Domestic cigarettes	26	10	10
21	46	—	Smoker	Domestic cigarettes	26	5	12

**Table 3:** fMRI brain response during left foot stimulation.

Patient no.	Right hemisphere						Left hemisphere							
	Postcentral gyrus of the parietal lobe	Precentral gyrus of the frontal lobe	Other parts of the frontal lobe	Others parts of the parietal lobe	Occipital lobe	Temporal lobe	Postcentral gyrus of the parietal lobe	Precentral gyrus of the frontal lobe	Other parts of the frontal lobe	Other parts of the parietal lobe	Occipital lobe	Temporal lobe	Postcentral gyrus of the parietal lobe	Precentral gyrus of the frontal lobe
1	Present with an intense signal		Present							Present				
3	Present with an intense signal		Present				Present			Present				Present
4	Present		Present							Present				
5	Present with an intense signal	Present	Present							Present	Present			Present
6	Present		Present	Present			Present	Present		Present	Present			
7	Present with an intense signal		Present							Present				
8	Present with an intense signal	Present	Present						Present	Present				
9	Present	Present												
10	Present with an intense signal		Present	Present						Present	Present			
11	Present with an intense signal	Present	Present							Present				
12	Present	Present	Present							Present				
13	Present with an intense signal		Present							Present				
14	Present with an intense signal	Present	Present						Present	Present				
15	Present with an intense signal	Present	Present							Present				
16	Present		Present	Present						Present				
17	Present with an intense signal		Present	Present						Present	Present		Present	
18	Present	Present	Present							Present	Present			
19	Present	Present								Present				
20	Present with an intense signal	Present	Present							Present	Present		Present	
21	Present with an intense signal	Present	Present		Present					Present	Present		Present	Present
														

**Table 4:** fMRI brain response during right foot stimulation.

Patient No.	Right hemisphere							Left hemisphere						
	Postcentral gyrus of the parietal lobe	Precentral gyrus	Other parts of the frontal lobe	Other parts of the parietal lobe	Occipital lobe	Temporal lobe	Thalamus	Postcentral gyrus of the parietal lobe	Precentral gyrus of the frontal lobe	Other parts of the frontal lobe	Other parts of the parietal lobe	Occipital lobe	Temporal lobe	Thalamus
1								Present	Present	Present				
3	Present		Present	Present		Present	Present	Present with an intense signal	Present	Present	Present		Present	Present
4	Present		Present						Present	Present				
5			Present					Present	Present with an intense signal	Present				
6	Present		Present	Present	Present	Present	Present	Present		Present	Present			Present
7	Present							Present		Present	Present			
8			Present						Present	Present				
9	Present	Present												
10								Present	Present	Present				
11			Present	Present				Present		Present	Present			
12			Present					Present with an intense signal	Present	Present				
13							Present		Present				Present	Present
14			Present					Present with an intense signal	Present					
15			Present					Present with an intense signal	Present	Present				
16								Present	Present					
17				Present				Present with an intense signal		Present	Present			
18			Present	Present					Present	Present	Present with an intense signal			
19			Present					Present	Present	Present				
20			Present					Present with an intense signal	Present	Present			Present	Present
21	Present		Present		Present	Present		Present with an intense signal	Present	Present	Present		Present	Present

## Data Availability

The fMRI raw data used to support the findings of this study have been deposited in the ResearchGate repository (DOI: 10.24203/ajas.v7i1.5743).
